The article "Alteration of Intestinal Microbiota and Hydrogen Sulfide Metabolism in Patients with Hashimoto's Thyroiditis" was retracted in 2023. Reasons: signs of a paper mill; compromised peer review; unreliable results or conclusions.

# Alteration of Intestinal Microbiota and Hydrogen Sulfide Metabolism in Patients with Hashimoto's Thyroiditis

**DOI:** 10.1155/2023/9302189

**Published:** 2023-07-10

**Authors:** Shangqing Zhang, Yan Chi, Hongfang Jin, Xiuli Wang, Xue Zhao, Ying Gao, Junqing Zhang

**Affiliations:** ^1^Department of Endocrinology, Peking University First Hospital, Beijing 100034, China; ^2^Department of Gastroenterology, Peking University First Hospital, Beijing 100034, China; ^3^Department of Pediatric, Peking University First Hospital, Beijing 100034, China

## Abstract

**Objective:**

To analyze the intestinal microbiota and H2S levels in patients with HT.

**Methods:**

Twenty euthyroid HT patients and twenty healthy control individuals were recruited. Fecal samples were collected, and the microbiota was examined using 16S RNA gene sequencing. We also collected serum samples to examine the H2S levels.

**Results:**

Compared with patients with HT, the ACE and Chao indices were significantly lower in healthy controls (*P*=0.04, 0.03, respectively). The microbial composition of the HT group differed significantly from that of the healthy group. We observed a significant increase in the proportions of *Bacteroides*, *Fusobacterium*, *Sutterella*, and *Veillonella* in patients with HT (*P* < 0.05). Linear discriminant analysis and effect size analysis also revealed that *Bacteroides* and *Ralstonia* were enriched in patients with HT. Additionally, patients with HT had significantly lower H2S levels than healthy controls (*P* < 0.005). The enrichment of H2S anabolism was linked to the alteration of intestinal microbiota in patients with HT.

**Conclusion:**

We demonstrated that patients with HT have aberrant intestinal microbiome and that H2S anabolism may contribute to HT pathogenesis.

## 1. Introduction

Hashimoto's thyroiditis (HT) is the chronic inflammation of the thyroid gland and is considered the most common autoimmune disease worldwide [1]. Clinically, HT is frequently asymptomatic. With the destruction of thyroid cells, patients with HT may develop subclinical or even overt hypothyroidism.

HT is related to an interaction of genetic elements, environmental factors, and epigenetic influences [2]. Dysbiosis of intestinal microbiota can trigger several immune disorders that are adjacent to or distant from the site of their induction [3]. Intestinal microbiota has also been considered to be involved in the pathogenesis of HT. In recent years, several studies have described the alteration of intestinal microbiota in patients with HT [4–8]. Emerging evidence has revealed that the dysbiosis of the intestinal microbiota is associated with the pathogenesis of Hashimoto's thyroiditis (HT). Hydrogen sulfide (H2S) is a metabolite of the intestinal microbiota that can regulate the viability and function of immune cells. However, the link between H2S and HT remains unclear. Changes in microbiota-derived metabolites, such as bile acids and short-chain fatty acids, also have regulatory effects on immune function. These changes in the corresponding metabolites can induce local or systemic inflammation [9]. Therefore, we further speculated that the levels of metabolites of the intestinal microbiota were different between patients with HT and healthy controls and that they may participate in the pathogenesis of HT.

Hydrogen sulfide (H2S), an endogenous product of bacteria and mammals, is the third gasotransmitter (along with nitric oxide and carbon monoxide) [10]. H2S can regulate the viability and function of immune cells. Downregulation of H2S leads to the development or worsens the severity of various immune-mediated diseases, including autoimmune rheumatoid arthritis and asthma [11, 12]. However, the relationship between H2S and HT remains unclear. H2S can also be produced by bacteria in the intestine. Depending on the microorganism, the production of H2S occurs in two ways: assimilatory sulfate reduction (ASR) and dissimilatory sulfate reduction (DSR). The only the terminal product of DSR is H2S [13]. Various gastrointestinal bacteria, especially sulfate-reducing bacteria (SRB), can produce exogenous H2S and regulate host H2S bioavailability and metabolism, consequently regulating physiological responses, such as epithelial cell health and inflammation [14]. Therefore, we speculated that the aberrant intestinal microbiota may downregulate the metabolism of H2S, which impairs immunoregulation and promotes the pathogenesis of HT.

In this study, we explored the differences in intestinal microbiome composition and serum H2S levels between patients with HT and healthy controls. We also analyzed H2S metabolism in the intestinal microbiota of patients with HT and healthy controls.

## 2. Materials and Methods

### 2.1. Patients and Samples

Twenty untreated euthyroid HT patients (19 females and one male), with an average age of 35.4 ± 9.4 years, were recruited from the Department of Endocrinology at the Peking University First Hospital from August 2020 to October 2021. The diagnosis of HT was defined as follows [15]: (1) highly elevated serum thyroid peroxidase antibody (TPOAb) and/or thyroglobulin antibody (TgAb) and (2) diffuse thyroid morphological features on an ultrasound examination. Twenty healthy volunteers (19 females and one male) with an average age of 33.9 ± 8.3 years old were recruited as controls. All controls were free of thyroid diseases based on an ultrasound examination and had no history or family history of thyroid diseases. These controls were euthyroid and negative for thyroid autoantibodies. All subjects with other autoimmune diseases or diseases that affected the intestinal microbiota based on the literature were excluded. Subjects treated with antibiotics, proton pump inhibitors, probiotics, or laxatives in the month before fecal sample collection were also excluded. Venous blood and fecal samples were collected from all subjects in the morning and stored at −80°C until use. This study was approved by the Ethics Committee of Peking University First Hospital (No. 2020-089) and conducted in accordance with the guidelines provided by the World Medical Association and the Helsinki Declaration. Informed consent was obtained from all the study subjects.

### 2.2. DNA Extraction from Human Fecal Samples

Total genomic DNA was extracted from human fecal samples using the CTAB/SDS method. The DNA concentration and purity were evaluated on a 1% agarose gel.

### 2.3. Polymerase Chain Reaction (PCR) Amplification

The V3-V4 hypervariable region of the 16S rRNA gene was amplified using the primers 515F (5′-GTG CCA GCM GCC GCG GTA A-3′) and 806R (5′-GGA CTA CHV GGG TWT CTA AT-3′). PCR reactions were conducted using Phusion® High-Fidelity PCR Master Mix (New England Biolabs). The PCR products were mixed in equidensity ratios and were agarose gel purified using the Qiagen Gel Extraction Kit (Qiagen, Germany).

### 2.4. Library Preparation and Sequencing

Sequencing libraries were generated using the TruSeq® DNA PCR-Free Sample Preparation Kit (Illumina, USA) following the manufacturer's recommendations, and index codes were added. Library quality was assessed using a Qubit® 2.0 Fluorometer (Thermo Scientific) and Agilent Bioanalyzer 2100 system. Finally, the library was sequenced on an Illumina NovaSeq 6000 platform, and 250 bp paired-end reads were generated.

### 2.5. Microbial Analysis

Paired-end reads were merged using overlapping sequences. Sequences were optimized by filtering and quality control. Operational taxonomic units (OTUs) were clustered using a 97% similarity cutoff with USEARCH (Version 11.0.667, https://www.drive5.com/usearch/), and chimeric sequences were identified and removed. The taxonomy of each sequence was annotated using the RDP Classifier (Release 11.1, https://rdp.cme.msu.edu/) in conjunction with the Silva database with a confidence threshold of 0.8. The *α* diversity was analyzed based on species richness at the OTU level, including the Chao, Shannon, ACE, and Simpson indices. Principal coordinate analysis (PCoA) based on Bray–Curtis dissimilarity was used to analyze structural differences between the samples using *ß* diversity. Linear discriminant analysis effect size (LEfSe) was conducted using a linear discriminant analysis (LDA) ≥ 4 to detect potential bacterial biomarkers. Statistical significance was set at *P* < 0.05.

PICRUSt software was used to predict the functional genes in the sequencing results, and functional classification was performed according to the Kyoto Encyclopedia of Genes and Genome (KEGG) database. We then analyzed the differences in the abundance of the two main metabolic pathways for H2S synthesis: M00176 (assimilating sulfate reduction pathway) and M00596 (dissimilatory sulfate reduction pathway).

### 2.6. Measurement of Serum H2S Levels by H2S Selective Sensor

H2S levels in serum samples were measured using the free radical analyzer TBR4100 with an H2S selective sensor (ISO-H2S-100, WPI, China), as previously described [16].

### 2.7. Statistical Analysis

GraphPad Prism (version 9.3.1) and R language 3.6.1 were used to process data, which are reported as mean ± standard deviation (SD). Student's *t*-test was used to compare the two groups. The Wilcoxon rank sum test was used to analyze the differences of the diversity index, microbiota abundance, and H2S metabolism pathway abundance between the two groups. Bivariate relationships were performed with a Pearson or Spearman rank correlation model. The Kruskal–Wallis rank sum test was used with LEfSe analysis. A *P* value < 0.05 was considered significant.

## 3. Results

### 3.1. Intestinal Microbiota Diversity and Composition in Patients with HT and Healthy Controls

Compared with the HT group, the ACE and Chao indices, which reflect abundance, were significantly lower in healthy controls (*P* = 0.04, 0.03, respectively) (Figures 1(a) and 1(b)). We analyzed *ß* diversity using Bray–Curtis principal coordinate analysis (Bray–Curtis PCoA). The results showed that the microbial composition of the HT group was significantly different from the healthy controls (Figure 1(e)). We determined the taxon composition of these two groups and sequenced 32 phyla and 596 genera. At the phylum level, the proportions of Bacteroidetes, Fusobacteria, and Tenericutes in patients with HT were significantly higher than those in healthy controls, and the proportion of Firmicutes in patients with HT was significantly lower (*P* < 0.05). At the genus level, the proportions of *Bacteroides*, *Fusobacterium*, *Sutterella*, and *Veillonella* in patients were significantly higher, and the proportions of *Blautia*, *Lachnoclostridum*, and *Roseburia* in patients were significantly lower (*P* < 0.05). (Figures 2(a) and 2(b)). We also identified specific bacterial taxa associated with the two groups using LEfSe analysis (linear discriminant analysis (LDA) > 4.0, all *P* < 0.05). At the genus level, *Bacteroides* and *Ralstonia* were enriched in patients in the LEfSe analysis. *Escherichia*, *Shigella*, *Blautia*, and *Faecalibacterium* were more enriched in the healthy controls (Figure 2(c)). The above results showed that patients with HT had aberrant intestinal microbiota.

### 3.2. H2S Levels in Serum Samples Were Lower in Patients with HT Compared to Healthy Controls

We found that H2S levels in serum samples from patients were significantly lower than those in healthy controls (*P* < 0.05) (Figure 3(a)). We also observed that the H2S was negatively correlated with the serum TgAb level (*r* = −0.533, *P*=0.0004, Figure 3(b)). This indicated that the alteration of the intestinal microbiota and downregulation of H2S were associated with HT.

### 3.3. H2S DSR Pathway Enrichment in the HT Intestinal Microbiota Was Downregulated

We analyzed the enrichment of the H2S metabolic pathway in the intestinal microbiota. There was no difference in the ASR between the two groups (Figure 3(c)). In DSR, the enrichment of intestinal microbiota from patients with HT decreased when compared to that of healthy controls (*P*=0.06, Figure 3(d)). This result suggested that the microbiota from patients with HT likely had a reduced ability to synthesize H2S.

## 4. Discussion

Several studies have discussed the causes of HT including genetic susceptibility and environmental factors. However, the pathogenesis of HT remains unclear [17]. Here, we verified that the intestinal microbiota in patients with HT differed from that in healthy controls. Patients with HT had lower H2S levels in the serum, and the metabolism of H2S in the microbiota from patients appeared to be downregulated.

Emerging evidence suggests that the intestinal microbiota is associated with the pathogenesis of HT. Several studies have described significantly different *ß* diversity in patients with HT compared with that in healthy controls [4–8]. A meta-analysis of the association between intestinal microbiota and autoimmune thyroiditis showed that the Chao index was increased in the HT group [18], which was consistent with our findings. The intestinal microbiota of patients was altered.

Our study showed that the incidence of *Blautia* was significantly lower in patients with HT. *Blautia* plays an important role in maintaining environmental balance in the intestine and preventing inflammation by upregulating intestinal regulatory T cells and producing short-chain fatty acids (SCFAs) [19]. The abundance of *Blautia* is negatively correlated with some inflammatory diseases [20]. Therefore, *Blautia* might be a protective bacterium genus from HT. The data showed that *Bacteroides* were enriched in patients with HT. *Bacteroides* is a pro-inflammatory bacterium that contributes to inflammatory bowel disease [21]. A study by Ishaq et al. also showed augmented *Bacteroides* levels in patients with HT [7]. The altered composition of the beneficial and harmful bacteria might be a possible factor in the pathogenesis of HT.

In addition to discussing the alteration of microbiota, we explored the mechanism by which microbiota affects thyroid autoimmunity. Immune cells are targets of H2S. T cell differentiation and function are significantly regulated by H2S [22]. The dysfunction of T cells, such as Th1, Th17, and regulatory T cells, is associated with the pathogenesis of HT [23–25]. There are no studies about the relationship between H2S and HT, to the best of our knowledge. Our results showed that H2S levels in the serum of patients were lower than those in healthy controls.

The intestinal microbiota can reduce sulfide to produce H2S and subsequently diffuse the H2S through the mucous membranes [26]. The reduction of H2S occurs by two pathways: ASR and DSR. Only the terminal product of DSR is H2S [13]. In our study, the enrichment of DSR in the intestinal microbiota decreased in patients, and this may be attributed to the downregulation of serum H2S levels in patients with HT.

We analyzed the intestinal microbiota in untreated euthyroid HT patients to avoid the influence of different thyroid functions and medications on intestinal microbiota. Our study is the first to explore H2S levels in patients with HT. However, our study does have some limitations. First, a relatively small number of participants were enrolled in the fecal microbiota analysis. Despite the small sample size, this study confirmed alterations in the intestinal microbiota. Secondly, a decreasing trend was observed in the enrichment of the HT intestinal microbiota of the DSR pathway, which may be related to the small number of participants.

## 5. Conclusion

In summary, our study demonstrated an altered intestinal microbiota and downregulated H2S metabolism in patients with HT. Alterations in the intestinal microbiota and H2S metabolism may be a novel mode of HT pathogenesis.

## Figures and Tables

**Figure 1:** *α* and *ß* diversity of the intestinal microbiota in patients with HT and healthy controls. (a–d) Microbial *α* diversity in patients with HT and healthy controls. The richness was significantly lower in healthy controls according to the ACE and Chao indexes. (e) Microbial *ß* diversity. Bray–Curtis principal coordinate analysis (Bray-Curtis PCoA) revealed that the microbial composition in patients with HT differed from that in healthy controls. ^*∗*^*P* < 0.05. HT, Hashimoto's thyroiditis.

**Figure 2:** Altered composition of intestinal microbiota in patients with HT and healthy controls. (a) Composition of the intestinal microbiota at the phylum level. (b) Composition of the intestinal microbiota at the genus level. (c) The LEfSe was used to identify species that significantly differed between patients with HT and healthy controls (LDA score of >4 and a significance of *P* < 0.05). HT, Hashimoto's thyroiditis.

**Figure 3:** Serum levels of H2S and the metabolism of H2S in intestinal microbiota. (a) The serum levels of H2S in patients with HT and healthy controls. (b) The correlation between H2S and TgAb. (c) The richness of the ASR pathway in intestinal microbiota from two groups. (d) The richness of the DSR pathway in intestinal microbiota from two groups. ^∗∗∗^*P* < 0.05. ASR, assimilatory sulfate reduction; DSR, dissimilatory sulfate reduction; HT, Hashimoto's thyroiditis; TgAb, thyroglobulin antibody.

## Data Availability

The data used to support this study are available from the corresponding author upon request.
